# 3D Animation Automatic Generation System Design Based on Deep Learning

**DOI:** 10.1155/2022/1434599

**Published:** 2022-06-09

**Authors:** Yongli Cao, Lei Wan, Lili Shi

**Affiliations:** Qingdao Huanghai University School of Arts, Qingdao, Shandong Province 266400, China

## Abstract

In the field of 3D animation design and generation, the expression generation method of animation is not obvious due to the lack of image details, which leads to the lack of realism of the generated animation expressions. In order to solve this problem, a deep learning-based animation character expression generation method is proposed. The method, based on the real facial expression images, uses improved deep learning to design cascade classifiers, extracts facial expression feature images from real images, softens image edges, and enhances feature details. The content and style of images are unified, the loss function is designed from the content constraints and style constraints, the judgment network is optimized, and the feature information is fused under the constraints of the loss function to generate the facial expressions of animated characters. The experimental results show that the design based on the feature point location of the improved deep learning expression generation method is accurate, the Pearson correlation coefficient between the input image and the generated image is high, the root mean square error is small, and the realism of the generated facial expression is enhanced.

## 1. Introduction

At present, deep learning technology has been successfully applied in many fields in the past ten years of research due to its very promising prospects. It has achieved good application results in various domains. Analysis of previous research results shows that, before deep learning technology is applied to a new field, it needs to continuously improve its own functions to make it more adaptable to new application backgrounds and better put into practical applications [1]. In the process of image processing, 3D animation character face generation is a new and very interesting research. Because 3D animation character face has a variety of expressions, it is widely welcomed by people, so many companies begin to use 3D animation style. As an image endorsement, people also use animated images on social platforms as their avatars on social platforms. Not only that, more and more 3D animation works have emerged in society [2–4]. It can be seen that the design of 3D animation characters has a very important position in the creation of animation works.

In the design and characterization of 3D animated characters, flexibility of facial expressions is an important content to show the characteristics of 3D animated characters and, thus, to enhance authenticity of the whole 3D animated characters [5]. The facial expression generation of 3D animation characters relies on the facial expression features of real faces, and the generation process is relatively complicated [6]. Through years of research by researchers and technical experts, a great breakthrough has been made in the processing of animation stylization, and it has been developed to date. A well-known mechanism, such as the animation expression generation method based on the improved CycleGan model mentioned in the literature [7], uses the CycleGan model and adopts the training form of subregions and weights the training results of the model to obtain the final facial expression image. However, there is a problem of blurred image details in the facial feature dataset, and the realism of the image is insufficient. In [8], a facial expression generation method based on improved conditional generation countermeasure network is proposed, but the problem of insignificant image details in practical applications has not been solved.

Therefore, an improved deep learning-based facial expression generation method for animated is proposed to address the aforementioned issues which are likely to occur if existing models are used. We have aimed to make full use of the enhanced deep learning technology to solve the problems existing in the above conventional facial expression generation methods.

The rest of the paper is organized as presented as follows. In section entitled “Design of 3D animation generation method based on deep learning,” a detailed description of the deep learning-based 3D animation generation methods, has been presented along with thorough analysis. Additionally, supportive mathematical equations of different parameters are also reported. Likewise in section entitled “experimental research on facial expression generation method of animated characters based on improved deep learning,” experimental setup along with how the proposed model is used on the real time dataset to resolve the problem at hand. Finally, concluding remarks are given.

## 2. Design of 3D Animation Generation Method Based on Deep Learning

### 2.1. 3D Animation Feature Extraction Based on Improved Deep Learning

Before generating the facial expressions of 3D animated characters, the real facial expression images are used as the basis for generating animation expressions. Before extracting the facial expression features of the real images, grayscale conversion is used for images with different attributes to unify the image attributes [9], and then improved deep learning is used to extract concave facial expression features. The improved deep learning technology has the distinguishing ability in the extraction of facial expression features. The improved deep learning technology is used to process real facial expression images, extract facial features from them, and use them as the basis for generating 3D animated character expressions. An image includes multiple units. Before processing, the image is divided into multiple blocks in units. Each block corresponds to a subarea, which is represented as A24–A, and the corresponding histogram is extracted from each subarea. The calculation is performed as shown in the following formula:

(1) $$\begin{array}{c} g_{i,j}=\sum_{x,y}p\left(\left(x,y\right)\in A_{i}\right). \end{array}$$

In the formula, *i* ∈ [1, *n*], *j* ∈ [1, *n*], *x*, and *y* represent image pixels and *g*_0_ represents the histogram in the ith subregion. The total histogram *G*_*A*_=(*g*_*i*,0_, *g*_*i*,1_,…, *g*_*i*,*n*_) is formed by the connection of the histograms of each subregion, which is used as the real facial expression feature sequence in the article.

When detecting the facial expression features of real faces, a cascade classifier is constructed by using deep learning technology. These classifiers are used to detect the real facial features of the input people at multiple scales. Multiscale detection is mainly aimed at images with more pixels. Before detecting features, a cascade classifier is trained. Based on the size of the input image [10–12], the search window is initialized and processed, and the search window is continuously trained according to the changes of the input image. Search for face features and merge the same face feature regions together. After the search is completed, a large number of subwindows are output, the images are filtered through the cascade classifier, a judgment is made at each node whether to discard the area, and finally a reasonable 3D animation expression feature set is obtained.

When the cascade classifier detects 3D animated facial expression images, the image size is not fixed. In order to improve work efficiency [13], use the nearest neighbor difference to adjust the size of the image. When the image processing operation is to enlarge, it may lead to increased aliasing of the image and hard image edges. Use the antialias method to soften the image edges and increase the realism of the image edges. Then, the pixels of the 3D animation image are normalized to obtain reliable and complete facial expression features.

### 2.2. Design Loss Function

In order to ensure that the facial expression details of the generated 3D animation are consistent with the real facial expression details [14], the style and content of the generated expression images are constrained. Assuming that the set of real facial expression images is *I*, the set of animated character expression images is *C*, and the input images are *x* ∈ *I*, *y* ∈ *Cx* EI, *y*, EC, the generated facial expression images are *J*(*K*_*t*_(*x*), *K*_*s*_(*y*)) denoted by *f*, where *J* denotes the decoder, *k* is the content encoder, and *k* is also the style encoder. Assuming that the input 3D animation feature image has two scales, let the outputs of the two scales be *Z*_1_ and *Z*_2_, and the output of the improved deep learning discriminant network is *Z* and *xZz*; then, the loss of the discriminant network is as shown in formulas (2) and (3):

(2) $$\begin{array}{c} \phi =1-Z_{1}\left(ff\right)*Z_{2}{\left(ff\right)}^{2}, \end{array}$$

(3) $$\begin{array}{c} \phi_{s=\frac{1}{2}}\left[\left(1-Z_{1}{\left(y\right)}^{2}\right)+\left(Z_{1}{\left(ff\right)}^{2}\right)\right]+\frac{1}{2}\left[\left(1-Z_{2}{\left(y\right)}^{2}\right)+\left(Z_{2}{\left(ff\right)}^{2}\right)\right]. \end{array}$$

In the case of unpaired data, the constraints on content are difficult to achieve through real facial expressions. Therefore, the form of reconstruction is used to ensure that the content of the expression image remains unchanged. The reconstruction process of the expression image is shown in Figure 1.

Input the human image *x*, and fuse its own content features with the real face expression style features to obtain the reconstructed image, which is recorded as *rec*_*x*1. In order to keep the content unchanged, in the reconstruction process, it is necessary to ensure that the generated 3D animated facial expression image is consistent with the original image content as much as possible, fuse it with the style features of the real facial expression image, and mark the obtained reconstructed image as *rec*_*x*2. The calculation formula for the two images is as shown in formulas (4) and (5):

(4) $$\begin{array}{c} rec\_x1=J\left(K_{t}\left(x\right),K_{s}\left(z\right)\right), \end{array}$$

(5) $$\begin{array}{c} rec\_x2=J\left(K_{t}\left(ff\right),K_{s}\left(z\right)\right). \end{array}$$

In the above formula, *z* represents an image with a similar style to the input image. In order to ensure the consistency of content and style between the reconstructed image and the input image, the *L*_1_ loss function in deep learning is used to constrain the expression image, which is used as the judgment network. The basis of the content loss is as shown in the following formula:

(6) $$\begin{array}{c} \left\{\begin{array}{c} L_{1}={\left\|x-rec\_x1\right\|}_{1},\\ L_{2}={\left\|x-rec\_x2\right\|}_{2}. \end{array}\right. \end{array}$$

In order to keep content of the expression image unchanged and retain the detailed features, equation (5) is used to constrain the content loss of the expression image. With support, you can adjust the weight to realize the constraints on the expression content. The specific contents as shown in the following formula:

(7) $$\begin{array}{c} L=\alpha_{1}L_{1}+\alpha_{2}L_{2}. \end{array}$$

The obtained loss function is used for the optimization of the generation network and discriminant network for generating facial expressions of animated characters. After the optimization is completed, based on the designed loss function, the facial expressions of animated characters are generated by improving deep learning.

### 2.3. Generate 3D Animated Character Facial Expressions

To generate facial expression images of 3D animated characters, it is necessary to use the extracted real facial expression features, fuse multi-angle facial expression feature maps [15], and obtain face feature information to realize the generation of various facial expressions of 3D animated characters.

The facial information of real faces contains different angles. Since the feature information of the same face at different angles is similar [16], similar pixel values represent the overall features of the face, and only a small number of different pixels represent the facial features of the face at a certain angle. . When calculating the pixel weight of each feature map, the parameter of the jump degree between pixels is introduced, and the pixel weight is represented by the jump degree more completely.

When calculating the weight of the feature map, the angle weight of the facial expression feature image of the 3D animation face is represented by a normal distribution, and the mean value of the normal distribution is limited to 0. After inputting *n* real face feature maps [17], calculate each feature map. The jump degree of each pixel is multiplied by the calculation result and the angle weight to obtain the overall weight of the image. After the feature fusion is completed, the facial expression of the 3D animated character is obtained calculated as follows:

(8) $$\begin{array}{c} x\left(p_{i}\right)=\frac{1}{\sqrt{2\pi \sigma }}\exp\left(-\frac{{\left(p_{i}-u\right)}^{2}}{2\sigma^{2}}\right),\\ \left|I_{m-1,n}+I_{m,n-1}+I_{m+1,n}+I_{m,n+1}-4*I_{m,n}\right|,\\ k_{i}\left(m,n\right)=x\left(p_{i}\right)*E_{i}\left(m,n\right),\\ h_{i\;d}=\frac{\sum {}_{i=1}^{n}k_{i}\left(m,n\right)\cdot h_{i\;d}\left(v_{pi}\right)}{\sum {}_{i=1}^{n}k_{i}\left(m,n\right)}. \end{array}$$

In the above formula, *σ* represents the decreasing degree of facial features, *V* represents the pixel value in the facial expression feature image, *x*(*p*_*i*_) represents the angle weight of image *i*, *E*_*i*_(*m*, *n*)represents the *n*-th row of image *i*, that is, the jumping degree of pixels in column *n*, *K*_*i*_(*m*, *n*) represents the overall weight of feature fusion *h*, and *a* represents the normalized processing result, ensuring that the pixel weight and weight sum are 1. After the feature images are fused and normalized, the resulting images are the facial expressions of animated characters.

So far, the design of the facial expression generation method for animated characters based on improved deep learning is completed.

## 3. Experimental Research on Facial Expression Generation Method of Animated Characters Based on Improved Deep Learning

### 3.1. Experimental Dataset

In the experimental research, the research on the facial expression generation method of 3D animated characters needs to convert from real face images to animated images and prepare 100 animated face images, which correspond one-to-one with the images in the face database. Considering the proposed face, the expression generation method uses deep learning techniques in the design. Before the experiment, two parts of data were screened from the original data set [18], one part of the data was used as the training set and the other part was used as the test set, and the two sets of data sets were recorded as data1 and data2, respectively. Similarly, the animation face dataset is also processed in the same way [19], and at the same time, all images used in the experiment are guaranteed to be 515 × 512 in size.

When studying the facial expression generation method of 3D animated characters, in addition to converting the real facial expressions into 3D animated expressions, it is also necessary to identify and locate the key points on the human face. Therefore, in the experimental design, the facial expression feature location experiment and the facial expression direction feature matching experiment are used to analyze the practical application effect of the facial expression generation method.

In order to avoid the incomplete facial expression feature image in the experiment, the blank boundary existing in the original image is filled before the experiment, and each filling takes a random form. The proposed facial expression generation method uses improved deep learning. After obtaining the experimental data [20], the experimental data are trained from end to end. The data training requires hardware with strong computing power as support. In the experimental research, the pytorch deep learning framework is used as support.

This experiment is mainly based on comparative experiments. After reading a large number of research materials, two more conventional expression generation methods are selected as reference, namely, the expression generation method of 3D animation based on the improved CycleGan model and the expression generation method based on the improved conditional generative adversarial network. For these two expression generation methods, the same experimental conditions are set to avoid other interference factors in the experiment from affecting the experimental results. After the experimental data set is prepared, the actual application effect of each method is verified.

### 3.2. Experiment Results of 3D Animation Facial Expression Feature Localization

In the facial expression feature localization experiment, the face data are annotated in the form of annotation, mainly focusing on three parts: body shape, hands, and legs. Considering the security of personal information, the key of each generation method is displayed on the 3D model, and the actual performance of each generation method is more intuitively compared and analyzed. The experimental results are shown in Figure 2.

Taking body shape, hand, and leg features as a reference and comparing the results in the observation figures, it can be seen that in the three sets of experimental results, the proposed method for generating facial expressions is more accurate in positioning the body shape, hand, and leg features, and there is no localization. In the case of point offset, the anchor point is concentrated at the set facial feature. In contrast, the other two groups of experimental results have more or less positional deviation, in which the positioning of the hand position has a relatively large deviation angle. Positioning information: the position of the legs and the position of the mouth are shifted downward, and the contour of the face is biased to the inside, and the overall positioning effect is not ideal. To sum up, the proposed method for generating facial expressions of 3D animated characters based on improved deep learning has better localization effect.

### 3.3. Experiment Results and Analysis of 3D Animation Facial Expression Feature Matching

Randomly select test samples from the test set in the prepared experimental data set, set a certain proportion of occlusion according to the experimental conditions, and use different expression generation methods to identify the test sample data in the data set. Expression comparison is used to judge the recognition level.

In the experiment, two objective indicators are used to measure different generation methods. The first indicator is the root mean square error, which is used to reflect the difference between the real face data and the generated data. The calculation formula is as follows:

(9) $$\begin{array}{c} RMSE=\sqrt{\frac{\sum {}_{i=1}^{n}{\left(y_{i}-y_{n}\right)}^{2}}{n}}. \end{array}$$

In formula (9), *y* represents the 3D animation expression feature data generated by the expression generation method, *y* represents the actual real facial expression data, and *i* represents the number of samples from 1 to *n*. The second experimental indicator is the Pearson correlation coefficient, which is calculated as follows:

(10) $$\begin{array}{c} w=\frac{\sum {}_{i=1}^{n}\left(y_{i}-y\right)\left(y-y_{i}\right)}{\sqrt{\sum {}_{i}^{n}\left(y_{i}-y^{\prime }\right){\left(y^{\prime }-y_{i}\right)}^{2}}}. \end{array}$$

In formula (10), *y*′ and *y*′ represent the mean value of *y* and *y*′, respectively, and *W* is the Pearson correlation coefficient, which represents the directional feature between the generated 3D animated facial expressions and the real facial expressions. If the value of *w* is close to 1, it means that the directional features between the two are infinitely close; on the contrary, if the value of *w* is close to 0, it means that the generated facial expression features have unsmooth jagged information, and the directional feature gap between the two is large. The experimental results are shown in Table 1.

From the data shown in Table 1, it can be seen that in the facial expression feature matching, the root mean square error of the proposed facial expression generation method is small, the Pearson correlation coefficient is close to 1, and the generated facial expression features are more similar to the real expression features. Facial expression feature matching is more accurate. The other two sets of experimental results show that with the increase in the occlusion area, the root mean square error becomes larger and larger and the Pearson correlation coefficient becomes smaller and smaller, approaching 0. It shows that when the original facial expression features are occluded, the facial expression features of the generated 3D animation are lost, and the expression images are incomplete. On the whole, the Pearson correlation coefficient of the proposed facial expression generation method based on improved deep learning is high, and the feature matching is more accurate. The root mean square error is small, and the realism of the generated 3D animated facial expressions is enhanced.

## 4. Conclusion

Due to its overwhelming characteristics, deep learning has been widely used in various research domains. From current research trend, deep learning technology has very good application prospects. In this paper, we have considered the autonomous generation of facial expressions of 3D animated characters as the main research content along with improving the progress of deep learning. We have designed a method for generating facial expressions of animated characters, which is based on deep learning, and localization experiment of 3D animation facial expression features is carried out to verify the operational superiority of the proposed model. Finally, through the matching experiments, it is proved that the proposed 3D animation facial expression generation method has a very good facial feature recognition effect. Additionally, generated facial expression features are more detailed, which has fully solved the problems associated with the traditional method and lay a solid foundation for the further development of the 3D animation design field.

## Figures and Tables

**Figure 1:** Reconstruction process of the expression.

**Figure 2:** Experimental results of body shape feature localization with different expression generation methods.

**Table 1:** Feature recognition experimental results of different 3D animation facial expression generation methods.

	Occlusion type	Block body type	Root mean square error	Pearson's correlation coefficient
Expression generation method based on improved CycleGAN model	Unobstructed	0 × 0	0.018	0.889
	Random block 25%	112 × 112	0.132	0.506
	Random block 50%	120 × 120	0.201	0.489

Expression generation method based on generative adversarial network	Unobstructed	0 × 0	0.305	0.968
	Random block 25%	112 × 112	0.425	0.669
	Random block 50%	120 × 120	0.021	0.589

The proposed expression generation method	Unobstructed	0 × 0	0.001	0.995
	Random block 25%	112 × 112	0.013	0.959
	Random block 50%	120 × 120	0.016	0.978

## Data Availability

The data used to support the findings of this study are available from the corresponding author upon request.
